The article "Design of Medical Image Detail Enhancement Algorithm for Ankle Joint Talar Osteochondral Injury" was retracted in 2023. Reasons: signs of a paper mill; suspected computer-generated content; unreliable results or conclusions; lack of ethics approval or compliance.

# Design of Medical Image Detail Enhancement Algorithm for Ankle Joint Talar Osteochondral Injury

**DOI:** 10.1155/2021/7381466

**Published:** 2021-10-29

**Authors:** Yundong Liu, Xufeng He

**Affiliations:** Affiliated Nanhua Hospital, University of South China, Health School of Nuclear Industry, Hengyang 421002, China

## Abstract

Medical imaging modalities, such as magnetic resonance imaging (MRI) and computerized tomography (CT), have allowed medical researchers and clinicians to examine the structural and functional features of the human body, thereby assisting the clinical diagnosis. However, due to the highly controlled imaging environment, the imaging process often creates noise, which seriously affects the analysis of the medical images. In this study, a medical imaging enhancement algorithm is presented for ankle joint talar osteochondral injury. The gradient operator is used to transform the image into the gradient domain, and fuzzy entropy is employed to replace the gradient to determine the diffusion coefficient of the gradient field. The differential operator is used to discretize the image, and a partial differential enhancement model is constructed to achieve image detail enhancement. Three objective evaluation indexes, namely, signal-to-noise ratio (SNR), information entropy (IE), and edge protection index (EPI), were employed to evaluate the image enhancement capability of the proposed algorithm. Experimental results show that the algorithm can better suppress noise while enhancing image details. Compared with the original image, the histogram of the transformed image is more uniform and flat and the gray level is clearer.

## 1. Introduction

Medical imaging modalities, such as magnetic resonance imaging (MRI) and computerized tomography (CT), have enabled clinicians and medical researchers to investigate the structural and functional features of the human body, thereby supporting the clinical diagnosis [1]. However, due to the highly controlled imaging environment (e.g., limited light intensities) of the human body, the imaging process often produces noise, which significantly affects the examination of the medical image. Therefore, signal denoising remains an important problem for the biomedical engineering community [2].

Due to the complexity of human body structure and tissues, and the influence of various factors such as X-ray scattering, electrical, and light quantum noise, X-ray medical images are characterized by wide dynamic range, large overlap, high noise, and poor contrast. At the same time, it is difficult for doctors to distinguish tissues and structures with a similar gray level when observing images. Clinicians not only understand the specific conditions of the patient's lesions based on the medical three-dimensional reconstructed model, but also use 3D printing and virtual reality technologies to achieve presimulation of the surgical site [3]. It also helps in reducing the surgical risk caused by doctors' subjective prediction, unclear preoperative doctor-patient communication, and unskilled operation. The effective processing of patients' original medical images before surgery (such as medical three-dimensional reconstruction, surgical path planning, and preoperative simulation exercises) has gradually become the development trend of surgical operations.

Image enhancement is the most basic technique in image processing technology [4]. Its main purpose is to enhance the useful information in the image, improve the visual effect of the image, according to the characteristics of the original image, purposefully enhance the overall or partial information of the image, and improve the original contrast and sharpness of the image, or the selective enhancement of some interesting details in the image while suppressing the uninteresting part of the image [5]. Meng and Qiao [6] presented a review of different techniques for medical image enhancement to improve the visual appearance of an image and highlighted various image enhancement methods for the medical professional. Cheng [7] proposed a mixed contrast enhancement technique for the improvement of the medical image that can provide a better solution to the image enhancement problems. Assessment has been done by signal-to-noise ratio, contrast-to-noise ratio, and Tenangrad measurement. It was reported that the proposed approach can provide better results than those of the adaptive enhancement and linear stretching; it is revealed that the proposed technique gives much better results than the existing ones. Sudhavani et al. [8] proposed a medical image enhancement technique of low-contrast images using fuzzy techniques. Three contrast enhancement techniques were presented based on fuzzy logic. In the first technique, the fuzzy system response function is implemented by simple if-then fuzzy rules. In the second method, the fuzzy contrast intensification operator is used as a method for improvement, and, in the third technique, the fuzzy expected value is employed as an image enhancement technique. Zhuang et al. [9] proposed an image enrichment method that includes several domains like classification, segmentation, and enhancement. Kaur and Kaur [10] used signal-to-noise ratio (PSNR), mean square error (MSE), normalization coefficient (NC), and root mean square error (RMSE) for enhancement of the medical images. Moreover, contrast enhancement is used to enhance the contrast of medical images. Issas and Kulkarni [11] presented a superresolution method for the enhancement of the medical images of the human body. A new image enhancement technique based on wavelet transform and Fourier series was presented by Bhardwaj and Singh [12]. Medical images were segmented with Haar transform followed by the decomposition of high-frequency subimages. The noise in the frequency field was decreased by applying the soft-threshold method. Next, the high-frequency coefficients were improved by different weight values of subimages. Then, the inverse Haar Transform was applied to obtain the enhanced image. Finally, the image's contrast was adjusted by nonlinear contrast enhancement methods. The method was effective for the enhancement of the image and was able to preserve the image edge to increase human visibility. Getreuer et al. [13] presented Automatic Color Enhancement (ACE) and its Fast Implementation for image enhancement. The algorithm was effective in improving the quality of images.

This paper proposes a new algorithm for the enhancement of the medical images of ankle joint talar osteochondral injury. The gradient operator is used to transform the image into the gradient domain, and fuzzy entropy is applied to replace the gradient to determine the diffusion coefficient of the gradient field. The finite differential operator is used to discretize the image, and the medical image partial differential equation enhancement model is constructed to achieve image detail enhancement.

The rest of the paper is organized as follows: In Section 2, an overview of the ankle osteochondral injury of the talus is presented.  Section 3 provides a detailed discussion of the proposed image enhancement algorithm. In Section 4, a case study is presented to elaborate the results of the proposed algorithm. Finally, the conclusion is given in Section 5.

## 2. Ankle Osteochondral Injury of the Talus

Most of the surface of the talus (about 60%) is covered by hyaline cartilage, without any attachment of muscles. The hyaline cartilage is mainly composed of collagen, proteoglycan, and water (high H+ content). The T1-weighted MRI shows isometric signals, and the T2-weighted fat pressure image showed a high signal. Cartilage lacks the characteristics of regeneration due to its lack of blood vessels, nerves, and lymphatic systems, and it lacks effective self-repair capabilities [13]. After damage, it is easy to cause osteochondrotis dissecans, subchondral bone cyst degeneration, and ischemic osteonecrosis.

Talar osteochondral injury is one of the important causes of ankle joint pain [14]. About 70% of the surface of the talus is covered by articular cartilage, and there is no muscle attachment. The blood vessels enter the talus in a concentrated position, and most of the talus is spongy bone, which can be injured by bone compression when it is traumatized and blood vessels in the bone. Therefore, damage to the cartilage of the talus can easily lead to a vascular necrosis of the talus.

In order to record the images of Talar osteochondral injury, we used the Skyra 3.0T magnetic resonance scanner from Siemens Germany for examination. The patient was instructed to lie in the supine position, with advanced feet. The MRI scanning ranged from the lower section of the tibia and fibula (including the inferior tibiofibular joint) to the level of the lower edge of the calcaneus. The scanning mode used was spin-echo sequence Tl-weighted image of lossy position, fast self-selected echo sequence (FSE) T2-weighted fat pressure image, coronal spin-echo sequence (SE) Tl-weighted image, and fast self-selected echo sequence (FSE) T2 fat pressure weighted image. The horizontal axis position fast self-selected echo sequence (FSE) T2 fat pressure weighted image and some PD weighted image sequences were added. The scanning parameters employed were layer thickness 3∼4 mm, layer spacing 0.5∼1 mm, matrix 256×256, and FOV 160 mm. The diameter, depth, and area of cartilage injury are shown in Figure 1.

The MRI findings were as follows: T1-weighted image of cartilage damage can clearly show uneven cartilage thickness, roughness, etc. and can also show the lack of integrity and displacement of the articular cartilage on the surface of the talus, and the increase of cartilage signal on T2-weighted image. In subchondral bone changes, the T1-weighted image shows a sheet-like low-intensity area with bone marrow edema in the subchondral bone of the talus, and the T2-weighted image shows high-intensity.

## 3. Medical Image Detail Enhancement Algorithm

In the process of medical image imaging, due to the influence of various factors, the images obtained by any medical imaging equipment will be interfered by noise to varying degrees and exhibit blurry details, low contrast, and poor visual effects. Medical image enhancement is to extract useful information in an image and suppress background information and noise through enhancement algorithms, improve the visual effect of the image, and help doctors diagnose and analyze the condition [15]. The image enhancement method of partial differential equation combines mathematical theories such as differential geometry, variational method, and functional analysis, which can effectively improve the contrast of the image and sharpen the image details. Image sharpening is mainly used to compensate for image contours, restore and enhance image details, and make the image clear, using its inverse operation form-differentiation to enhance the details and edges of the image.

### 3.1. Medical Image Enhancement Based on Partial Differential Equations

The gradient operator is used to transform the image into the gradient domain, and then the gradient field of the image is linearly stretched as the target contrast, and the image is reconstructed from the target contrast field by the variational method. The specific process of the algorithm is as follows:

Suppose that a gray image with *M* × *N* dimensions can be represented *I*=[*f*(*i*, *j*)]_*M*×*N*_,  (*i*, *j*) ∈ Ω={0 ≤ *i* ≤ *M* − 1,0 ≤ *j* ≤ *N* − 1}; then, the gradient *p* ∈ Ω at any point in the image can be defined as

(1) $$\begin{array}{c} \nabla I\left(p\right)=\left(\frac{\partial I}{\partial i}\left(p\right),\frac{\partial I}{\partial j}\left(p\right)\right),\;p\in \Omega . \end{array}$$

For an image, the direction of the gradient indicates the direction of change in the grayscale, and the size of the gradient indicates the speed of the grayscale change. The sum of the gradient size and direction of all pixels constitutes the gradient vector field of the image, that is, the contrast vector field.

To enhance the image, *I* is to find another image *I*′ so that the contrast field ∇*I*′(*p*) of the image *I*′ is satisfied: in terms of value, |∇*I*′(*p*)| > |∇*I*(*p*)| and the direction is consistent with ∇*I*(*p*). There is no doubt that the new image *I*′ will be visually clearer than *I*. This can be represented using the following mathematical equations:

(2) $$\begin{array}{c} T_{I{}^{\prime }\left(p\right)}=C\cdot T_{I\left(p\right)}\\ =\left\{\begin{array}{c} C\cdot \nabla I\left(p\right),\;\left|\nabla I\left(p\right)\right|>\varepsilon ,\\ 0,\;\left|\nabla I\left(p\right)\right|\leq \varepsilon , \end{array}\right. \end{array}$$

where *T*_*I*′(*p*)_ is the gradient field of the enhanced image. *ε* is the noise threshold, and it is considered that the gradient is smaller than *ε* that is caused by noise. The magnification of *C* contrast is generally *C* > 1, but the value of *C* cannot be too large; otherwise, the noise will be amplified.

In equation (2), if the magnification factor *C* is taken as a constant, then the method has the same contrast magnification at the strong edge and the weak edge, and the contrast enhancement of the weak edge of the image may not be obvious, and the phenomenon of the strong edge is overenhanced. In order to overcome this shortcoming, we construct a gradient-based amplification factor as

(3) $$\begin{array}{c} C\left(\nabla I\right)=1+\frac{\lambda }{1+{\left(\nabla I/k\right)}^{2}}, \end{array}$$

where *λ* represents the amplification factor and *λ* > 0*k* > 0 shows the speed at which the diffusion coefficient decreases as the gradient increases. It can be seen from equation (3) that the magnification factor decreases with the increase of the original image gradient value; that is, the magnification factor of high-contrast pixels is smaller, which avoids overenhancement. Low-contrast pixels have a larger magnification factor, which can effectively magnify small details that are not easily noticeable, so the enhanced image looks softer.

The image *I*′ is reconstructed from the stretched contrast field; that is, the image *g* is searched to minimize the functional of equation (4).

(4) $$\begin{array}{c} v\left(f\right)=\int \int_{\Omega }{\left|\nabla g-T_{I^{\prime }\left(p\right)}\right|}^{2}d\Omega ,\;g\left(p\right)|{}_{\forall p\in \Omega }, \end{array}$$

where *T*_*I*′(*p*)_ is the gradient field after reconstruction. Using the variational method to solve the following equation, the following Euler–Lagrange equation can be obtained:

(5) $$\begin{array}{c} \Delta g=\text{div}G. \end{array}$$

In equation (5), Δ represents the Laplace operator and has Δ*g*=(∂^2^*g*/∂*x*^2^)+(∂^2^*g*/∂*y*^2^). By solving the above equation, the enhanced image *g* can be obtained.

### 3.2. Introducing Fuzzy Entropy to Enhance Medical Image Details

The fuzzy gradient field is used to replace the gray domain gradient. Secondly, the fuzzy entropy is applied to replace the gradient to determine the diffusion coefficient of the gradient field. Entropy has an important physical meaning in information theory, and it is a physical quantity used to measure the degree of uncertainty in probability distribution [16]. Similarly, the concept of entropy can also be introduced in fuzzy set theory, called fuzzy entropy, to measure the degree of fuzzy set. The fuzzy entropy can reflect the spatial change rate of the image gray value, so it can distinguish the edge area and the smooth area of the image, and when the input image is noisy, the edge of the fuzzy entropy positioning is finer and more accurate [17].

Assume a digital image *I*=[*f*(*i*, *j*)]_*M*×*N*_ of size *M* × *N*, where *f*(*i*, *j*) represents the gray value of the (*i*, *j*) pixel. Take a window *W*_*n*_(*i*, *j*) whose center is (*i*, *j*) and size *n* × *n*. The gray matrix of the original image covered by this window is as follows:

(6) $$\begin{array}{c} W_{n}\left(i,j\right)=\left[\begin{array}{ccc} f\left(i-1,j-1\right) & f\left(i,j-1\right) & f\left(i+1,j-1\right)\\ f\left(i-1,j\right) & f\left(i,j\right) & f\left(i+1,j\right)\\ f\left(i-1,j+1\right) & f\left(i,j+1\right) & f\left(i+1,j+1\right) \end{array}\right]. \end{array}$$

Taking the grayscale matrix *W*_*n*_(*i*, *j*) as the domain of discourse, the equivalent fuzzy set $\tilde{A}$ of an image can be defined in the domain of discourse, and the membership function (that is, the mapping function) is

(7) $$\begin{array}{c} \mu_{m}\left(f\left(i+k,j+l\right)\right)=\frac{1}{1+\left|f\left(i+k,j+l\right)-m\right|/\alpha },\;-\frac{\left(n-1\right)}{2}\leq k,\;l\leq \frac{\left(n-1\right)}{2}, \end{array}$$

where *m* represents the eigenvalue of the fuzzy set $\tilde{A}$ and *μ*_*m*_(*f*(*i*+*k*, *j*+*l*)) represents the degree to which *f*(*i*+*k*, *j*+*l*) belongs to the fuzzy set $\tilde{A}$. It is not difficult to conclude from equation (7) that if the difference between *f*(*i*+*k*, *j*+*l*) and *m* is smaller, the degree of membership of the pixel is greater. Similarly, if the difference between *f*(*i*+*k*, *j*+*l*) and *m* is larger, the pixel membership is smaller; *α* is the control factor (usually a constant) to ensure 0.5 ≤ *μ*_*m*_(*f*(*i*, *j*)) ≤ 1.

In order to better understand the fuzziness of fuzzy sets, Figure 2 shows the relationship curve between the fuzziness $\tilde{A}$ and the value of membership.

When $\mu_{{\overset{⌣}{A}}_{i}}\left(x\right)$ is near to 1/2, the affiliation between *x* and $\tilde{A}$ is the least certain, and the ambiguity is the greatest. When $\mu_{{\overset{⌣}{A}}_{i}}\left(x\right)$ is closer to 1 or 0, it means that the higher or the lower the *x* belonging to $\tilde{A}$, the smaller the corresponding ambiguity. The fuzzy entropy of the image can be defined on the equivalent fuzzy set of the image:

(8) $$\begin{array}{c} e\left(\tilde{A}\right)=\frac{1}{n\times n}\sum_{k=-\left(n-1\right)/2}^{\left(n-1\right)/2}\sum_{l=-\left(n-1\right)/2}^{\left(n-1\right)/2}H_{m}\mu_{m}\left(f\left(i+k,j+l\right)\right). \end{array}$$

Fuzzy entropy reflects the severity of image gray changes; that is, it can quantitatively describe the degree to which a certain pixel belongs to the edge. Suppose that the amplification factor *C*(*C* > 1) that attenuates as the fuzzy entropy increases:

(9) $$\begin{array}{c} C\left(E\left(\tilde{A}\right)\right)=1+\frac{\lambda }{1+{\left(E\left(\tilde{A}\right)/\alpha \right)}^{2}}. \end{array}$$

In equation (9), $E\left(\tilde{A}\right)$ is the fuzzy entropy of the fuzzy set determined by the membership function on the image *I*, *λ* > 0 shows the amplification factor, so the maximum value of *C* is (1+*λ*), and *α* > 0 represents the attenuation speed of the amplification factor *C* as $E\left(\tilde{A}\right)$ increases.

Figure 3 shows that the curve of the magnification coefficient is changing with the fuzzy entropy. When the blur entropy is small, the gradient field magnification is larger; that is, the weaker the details, the greater the magnification, so it can well enhance the original unnoticeable details. When the blur entropy gradually increases, the magnification becomes smaller and smaller, and eventually it tends to 1, which avoids excessive enhancement of sharply changing edges, so that the enhanced image looks softer.

Laplace change of binary image function *F* is

(10) $$\begin{array}{c} \nabla^{2}f=\frac{\partial^{2}f}{\partial x^{2}}+\frac{\partial^{2}f}{\partial y^{2}}. \end{array}$$

The Laplacian edge sharpening is expressed as

(11) $$\begin{array}{c} g\left(x,y\right)=f\left(x,y\right)-\alpha \nabla^{2}f\left(x,y\right). \end{array}$$

Among them, the enhancement coefficient *α* determines the degree of enhancement of the image. If *αt* is smaller, the degree of image enhancement is smaller, and if *α* is larger, the degree of image enhancement is greater. To be suitable for image processing, this equation needs to be discretized. The second-order partial differential in the *x*-direction is defined as

(12) $$\begin{array}{c} \frac{\partial^{2}f}{\partial x^{2}}=f\left(x+1,y\right)+f\left(x-1,y\right)-2f\left(x,y\right). \end{array}$$

Similarly, the *y*-direction is given as

(13) $$\begin{array}{c} \frac{\partial^{2}f}{\partial y^{2}}=f\left(x,y+1\right)+f\left(x,y-1\right)-2f\left(x,y\right). \end{array}$$

Likewise, the discrete form can be approximated using

(14) $$\begin{array}{c} g\left(i,j\right)=f\left(i,j\right)-\alpha \left[f\left(i+1,j\right)+f\left(i-1,j\right)+f\left(i,j+1\right)+f\left(i,j-1\right)-4f\left(i,j\right)\right]. \end{array}$$

Only the discretized differential operator can be used in digital image processing [18]. The finite difference is a common method for the discretization of the differential operator. Firstly, the digital image is sampled at equal intervals with Δ*x*=1 and Δ*y*=1, and then the forward difference and backward difference are used to discretize the Laplace operator and divergence operator, respectively. After obtaining the corrected membership value *μ*′, the image is transformed from the fuzzy domain to the gray domain according to the inverse transformation to obtain an enhanced image.

(15) $$\begin{array}{c} f_{ij}=\mu_{ij}^{\prime }\cdot \left(f_{\max}-f_{\min}\right)+f_{\min}. \end{array}$$

Based on the above analysis, the specific implementation steps of the algorithm are as follows:

- The image can be mapped from the gray domain to the fuzzy domain according to the membership function defined in equation (11)
- The Sobel operator can be used to calculate the image gradient and determine the parameter *A*
- The fuzzy entropy of the image is calculated according to equation (8), and the fuzzy entropy and *α* are substituted into equation (7) to obtain the magnification coefficient *C*
- Equation (15) is used to calculate the revised membership value
- The pixel value of the enhanced image is calculated, as well as the modified membership value

Fuzziness is an inherent attribute of medical images due to several reasons [19]. First, information loss is unavoidable in the process of mapping three-dimensional human organs or tissues into flat images. Secondly, the grayscale of a grayscale image is gradually transitioned from black to white, and the human eye cannot accurately distinguish the specific gray level. The third is that the definition of the edges and details of the structural organization in the image is fuzzy.

These ambiguities are difficult to describe in classical mathematical language, so fuzzy theory came into existence. On the one hand, fuzzy theory can quantitatively express ambiguous information and features in medical images. On the other hand, the final receiver of image information is the human eye. The fuzzy system can effectively simulate some human behaviors, such as perception, judgment, and resolution. Therefore, the image enhancement model based on fuzzy theory can not only quantitatively describe the image features, but also match the visual mechanism of the human eye. Therefore, it can obtain high-quality medical images and help doctors diagnose the disease quickly and accurately [20].

## 4. Case Analysis

The medical imaging data used in this article are all taken from 3D Slicer. 3D Slicer is a free, open source and multiplatform software package widely used for medical, biomedical, and related imaging research. The Data Store of this software provides a large amount of patient imaging data for medical researchers to download and use. Data store is shown in Figure 4.

For the medical 3D model obtained by segmentation and reconstruction of the patient's original 2D image, further preoperative simulation work can also be completed in the 3D slicer. In this section, the medical three-dimensional model after reconstruction of the ankle joint talar osteochondral injury is used as the input of the preoperative simulation, and the demonstration experiment performed is the preoperative simulated bone window.

As an important method to measure image quality, objective evaluation is used to build a quantitative index based on the human visual perception system to measure the image quality by calculating the size of the comparison index. To measure the image quality in the proposed image enhanced algorithm, we employed three objective evaluation indexes, namely, signal-to-noise ratio (SNR) or peak signal-to-noise ratio (PSNR), root mean square error (RMSE), information entropy (IE), and edge protection index (EPI). Let *f* represent the input image of *M* × *N*, *g* represent the enhanced image, and the gray values of a pixel (*i*, *j*) are *f*(*i*, *j*) and *g*(*i*, *j*), respectively, and then the objective evaluation indexes are defined in the following section. The EPI can be expressed as

(16) $$\begin{array}{c} \text{EPI}=\frac{\sum \sum \left|f\left(i,j\right)-f\left(i,j+1\right)\right|+\sum \sum \left|f\left(i,j\right)-f\left(i+1,j\right)\right|}{\sum \sum \left|g\left(i,j\right)-g\left(i,j+1\right)\right|+\sum \sum \left|g\left(i,j\right)-g\left(i+1,j\right)\right|}, \end{array}$$

where EPI is the edge protection index. The larger the EPI, the better the edge protection of the image, and the better the image enhancement effect. Likewise, equation (17) is used to represent information entropy:

(17) $$\begin{array}{c} \text{IE}=-\sum_{m=0}^{L-1}p\left(m\right)\log_{2}\;p\left(m\right), \end{array}$$

where *p*(*m*) is the probability of occurrence of gray level *m*, *L* represents the maximum gray level of the image, and the information entropy reflects the amount of image information. Therefore, if IE is larger, it means that the image contains more detailed information, and the image enhancement effect is better. The signal-to-noise ratio (SNR) of the image can be expressed as

(18) $$\begin{array}{c} \text{SNR}=10\;\log_{10}\frac{\sum_{i-0}^{M-1}\sum_{j-0}^{N-1}g{\left(i,j\right)}^{2}}{\sum_{i-0}^{M-1}\sum_{j-0}^{N-1}{\left(g\left(i,j\right)-f\left(i,j\right)\right)}^{2}}. \end{array}$$

SNR describes the ratio of the effective component and the noise component in the image. If the SNR is larger, it means that the effective information is more, and the noise is smaller. Therefore, the noise in the image after enhancement is smaller.

To explain more objectively, this study quantitatively describes the enhancement effect of the proposed algorithm from the three perspectives: edge protection ability, noise suppression ability, and detail enhancement ability.  Table 1 shows the edge protection index (EPI), signal-to-noise ratio (SNR), and information entropy (IE) of different image enhancement methods to enhance the image. It can be seen from the table that the edge protection index (EPI = 0.546) of the proposed image enhancement algorithm is smaller than the Cheng algorithm (EPI = 0.582), indicating that the edge protection capability is slightly weaker than the Cheng algorithm, but the signal-to-noise ratio (SNR = 15.362) and information entropy (IE = 6.985) are significantly higher than the other two algorithms; this shows that the proposed algorithm can better suppress noise while enhancing image details. The result of histogram equalization processing is shown in Figure 5.

Through the histogram equalization process, the contrast of the original input image is enhanced, and the histogram distribution of the input image is changed to a “uniform” histogram distribution. The histogram of the transformed image is more uniform and flatter compared to the original image histogram, and the grayscale level is clearer.

## 5. Conclusion

Medical images are the information source and provide a base for clinical diagnosis. However, due to the influence of various factors, medical images often have problems such as low contrast, noise pollution, details, or blurred edges. Improving the contrast of the image and enhancing the important details and edges in the image will help improve the efficiency and accuracy of medical diagnosis. Therefore, the research of medical image processing and analysis is gradually receiving more attention. In this study, a detailed enhancement algorithm for medical images of ankle joint talar osteochondral injury is proposed. The gradient operator is used to transform the image into the gradient domain followed by fuzzy entropy to replace the gradient to determine the diffusion coefficient of the gradient field. The medical image partial differential equation enhancement model is developed to achieve image detail enhancement. The introduction of a fuzzy entropy algorithm can better suppress noise while enhancing image details. Compared with the original image, the histogram of the transformed image is more uniform and flatter, and the gray level is clear. Although the improved algorithm proposed in this study can achieve the purpose of parameter adaptive selection, there are still parameters that need to be manually set, and the optimal value is selected after repeated experiments, which is inconvenient for clinical application. Therefore, the selection of parameters needs to be further improved in future research.

## Figures and Tables

**Figure 1:** Diameter, depth, and area of cartilage injury.

**Figure 2:** The relationship curve between the fuzziness of $\tilde{A}$ and the value of membership.

**Figure 3:** Amplification coefficient and *H*_*m*_*μ*_*m*_(*f*(*i*+*k*, *j*+*l*)) change curve with fuzzy entropy. (a) The curve of *H*_*m*_*μ*_*m*_(*f*(*i*+*k*, *j*+*l*)) changing with *f*. (b) The curve of magnification coefficient changing with fuzzy entropy.

**Figure 4:** Data store.

**Figure 5:** The result of histogram equalization processing. (a) Grayscale image. (b) Equalized image. (c) Histogram of the grayscale image. (d) Histogram after equalization.

**Table 1:** Objective evaluation parameters of each algorithm of the MRI image.

	EPI	SNR	IE
Cheng algorithm [7]	0.582	12.808	5.014
ACE method [13]	0.515	11.321	5.214
Proposed method	0.546	15.362	6.985

## Data Availability

The data used to support the findings of this study are available from the corresponding author upon request.
